# Dysbindin Promotes the Post-Endocytic Sorting of G Protein-Coupled Receptors to Lysosomes

**DOI:** 10.1371/journal.pone.0009325

**Published:** 2010-02-19

**Authors:** Aaron Marley, Mark von Zastrow

**Affiliations:** Departments of Psychiatry and Cellular and Molecular Pharmacology, University of California San Francisco, San Francisco, California, United States of America; Thomas Jefferson University, United States of America

## Abstract

**Background:**

Dysbindin, a cytoplasmic protein long known to function in the biogenesis of specialized lysosome-related organelles (LROs), has been reported to reduce surface expression of D2 dopamine receptors in neurons. Dysbindin is broadly expressed, and dopamine receptors are members of the large family of G protein-coupled receptors (GPCRs) that function in diverse cell types. Thus we asked if dysbindin regulates receptor number in non-neural cells, and further investigated the cellular basis of this regulation.

**Methodology/Principal Findings:**

We used RNA interference to deplete endogenous dysbindin in HEK293 and HeLa cells, then used immunochemical and biochemical methods to assess expression and endocytic trafficking of epitope-tagged GPCRs. Dysbindin knockdown up-regulated surface expression of D2 receptors compared to D1 receptors, as reported previously in neurons. This regulation was not mediated by a change in D2 receptor endocytosis. Instead, dysbindin knockdown specifically reduced the subsequent trafficking of internalized D2 receptors to lysosomes. This distinct post-endocytic sorting function explained the minimal effect of dysbindin depletion on D1 receptors, which recycle efficiently and traverse the lysosomal pathway to only a small degree. Moreover, dysbindin regulated the delta opioid receptor, a more distantly related GPCR that is also sorted to lysosomes after endocytosis. Dysbindin was not required for lysosomal trafficking of all signaling receptors, however, as its depletion did not detectably affect down-regulation of the EGF receptor tyrosine kinase. Dysbindin co-immunoprecipitated with GASP-1 (or GPRASP-1), a cytoplasmic protein shown previously to modulate lysosomal trafficking of D2 dopamine and delta opioid receptors by direct interaction, and with HRS that is a core component of the conserved ESCRT machinery mediating lysosome biogenesis and sorting.

**Conclusions/Significance:**

These results identify a distinct, and potentially widespread function of dysbindin in promoting the sorting of specific GPCRs to lysosomes after endocytosis.

## Introduction

G protein-coupled receptors comprise the largest family of signaling receptors expressed in animal cells, and control a vast array of physiological processes [1]. A fundamental determinant of cellular responsiveness to a particular GPCR-mediated extracellular stimulus is the number of cognate receptors present in the plasma membrane. Mammalian cells typically express multiple GPCRs responsive to distinct ligands, and it is thought that surface expression of particular GPCRs is regulated in a receptor-specific and ligand-dependent manner, allowing cells to dynamically regulate their responsiveness to particular ligands. Biochemical mechanisms that mediate such receptor-specific regulation of surface receptor number are thus of fundamental physiological importance.

In addition to their broad significance to normal physiology, GPCRs represent the single largest class of clinically relevant drug targets. Further, it is thought that disturbances in the function or expression of particular signaling receptors may contribute to a variety of pathological states [2]. The dopaminergic hypothesis of schizophrenia, for example, postulates that there is relative excess of signaling specifically via D2-type dopaminergic GPCRs in the brain [3]. Consistent with this, many of the drugs effective in the treatment of schizophrenia are selective D2 receptor antagonists. Schizophrenia is highly heritable but its genetics are complex. Of the various genes implicated in schizophrenia disease risk, a remarkable fraction encode proteins that function in membrane traffic [4]. Might human disease genetics provide new insight relevant to the membrane trafficking of specific GPCRs?

Recent data suggest that this may indeed be the case. Dysbindin, a cytoplasmic protein encoded by DTNBP1 [5], has been genetically linked to the Hermansky-Pudlak syndrome (HPS). HPS is characterized by hypopigmentation and bleeding problems resulting from loss of lysosome-related organelles, which are present in specialized secretory cell types such as melanocytes and platelets [6], [7], [8]. Interestingly, dysbindin has also been implicated more recently as a schizophrenia risk gene [9], [10], [11]. Dysbindin produces significant effects on dopaminergic signaling [12] and has been reported to reduce surface expression of D2 receptors, relative to the closely related D1 dopamine receptor in neurons [13].

Dysbindin is expressed widely in mammalian tissues [5], not only in specialized secretory cells. Further, dopamine receptors are expressed outside of the nervous system, and are members of the largest group of GPCRs (family A) that are expressed in many cell types. These considerations raise the question of whether dysbindin may also affect GPCR trafficking outside of the nervous system. We investigated this possibility in the present study. Here we show that dysbindin-dependent regulation of surface receptor expression is not restricted to neurons or to the D2 receptor, and identify an apparently widespread function of dysbindin in regulating GPCRs by promoting their sorting to lysosomes after endocytosis.

## Results

### Dysbindin Regulates D2 Receptor Number Observed at Steady State in the Plasma Membrane of Non-Neural Cells

To begin to investigate whether dysbindin functions in nonspecialized cell types, we used HEK293 cells as a model. Immunoblotting clearly detected endogenous dysbindin expression in these cells, and 3 different siRNAs targeting the human DTNBP1 gene effectively depleted endogenous dysbindin, with equivalent loading verified by blotting for GAPDH (Fig 1A). We then asked if dysbindin depletion affects surface expression of dopamine receptors in these cells. To do so we prepared stably transfected cells expressing FLAG epitope-tagged versions of either the human D1 or D2 dopamine receptor, and selected cell clones expressing similar amounts of receptor in the plasma membrane as assessed by fluorescence flow cytometry. siRNA-mediated knockdown of dysbindin significantly up-regulated FLAG-D2 receptor surface expression, but did not detectably affect surface expression of FLAG-D1 receptors (Fig 1B). We verified this effect (and the subsequent effects described), using all three (non-ovelapping) siRNA target sequences.

**Figure 1:** Dysbindin knockdown increases surface expression of recombinant D2 dopamine receptors in HEK293 cells. **A.** Immunoblot showing depletion of endogenous dysbindin in HEK293 cells by three different siRNA duplexes. A representative immunoblot is shown of cell extracts (30 µg/lane) from control-transfected (CTL) cells and cells transfected with one of three siRNA specific duplexes; similar results were obtained with each of the silencing duplexes The immunoreactive band corresponding to endogenous dysbindin is indicated by arrow. A small amount of cell extract (∼2 µg) from cells transfected with HA-DYS was run alongside to verify this assignment (right lane, HA-DYS resolves at a slightly higher apparent molecular mass then that endogenous protein due to the presence of the epitope tag). The high molecular band observed between the 160 and 260 kDa markers represents a nonspecific band useful for verifying comparable loading. GAPDH blot is shown in the panel below to further verify equivalent loading. **B.** Effect of dysbindin knockdown on relative surface receptor immunoreactivity of stably transfected HEK293 cells expressing either FLAG-D2R or FLAG-D1R (indicated by D2 and D1, respectively). Surface receptor immunoreactivity was determined by anti-FLAG labeling of intact cells and fluorescence flow cytometry, as described in *Materials and Methods*, comparing mean fluorescence values measured from cells transfected with the non-silencing control RNA duplex (CTL) and a silencing duplex (siRNA #1 from panel A). For each experiment, surface receptor immunoreactivity measured in cells transfected with the dysbindin-silencing duplex (DYS) was normalized to that measured in parallel determination from cells transfected with the non-silencing control duplex (CTL). Bars represent determinations averaged over multiple (≥5) experiments and the error bar indicates S.E.M. p values were calculated from the non-normalized individual data using a paired Student's t-test.

### Dysbindin Selectively Affects Trafficking of D2 Receptors to Lysosomes after Endocytosis

Selective up-regulation of surface D2 receptors observed in HEK293 cells is consistent with results reported previously from dysbindin knockdown in cortical neurons, which proposed that dysbindin is specifically required for endocytosis of D2 receptors. Thus we applied fluorescence flow cytometry to assess internalization of D2 receptors induced by addition of 10µM dopamine to the culture medium. Surprisingly, despite its pronounced effect on basal surface expression, dysbindin depletion in HEK293 cells did not detectably affect the rate or extent of FLAG-D2 receptor internalization (Fig 2A and B).

**Figure 2:** Dysbindin knockdown specifically inhibits proteolysis of internalized D2 receptors without detectably inhibiting receptor internalization. **A.** Flow cytometric analysis of dopamine-induced internalization of D2 dopamine receptors. Stably transfected HEK293 cells expressing FLAG-D2R, exposed for the indicated time periods to 10 µM dopamine, were analyzed by surface antibody labeling and flow cytometry. Loss of surface receptor immunoreactivity was used to assess ligand-induced internalization in cells transfected with dysbindin siRNA (DYS) and compared to cells transfected with a non-silencing control duplex (CTL). Points represent averaged values (normalized to cells not exposed to dopamine (t = 0) from ≥5 experiments and error bars indicate S.E.M. **B.** Fractional internalization measured after exposure cells to 10 µM dopamine for 30 min, showing the lack of significant difference between CTL and DYS conditions. **C.** Surface biotinylation experiment showing that dysbindin knockdown inhibits dopamine-induced proteolysis of FLAG-D2Rs. **D.** Quantification of time-dependent loss of surface-biotinylated FLAG-D2R in cells incubated for the indicated time period after surface biotinylation in the presence of 10 µM dopamine. **E.** Comparison of D2R degradation measured at the 4 hour time point over multiple experiments (n = 8), verifying the statistical significance (p = 0.001 by Student's t-test) of the observed inhibition. **F.** Biotin protection-degradation assay showing that dysbindin knockdown specifically inhibits degradation of D2Rs after internalization.

The failure of dysbindin depletion to affect D2 receptor internalization raised the question of whether the observed increase in steady state surface expression occurs via the endocytic pathway at all. To investigate this, we applied surface biotinylation to specifically label the plasma membrane pool of D2 receptors and assessed turnover of this receptor pool as a function of time. Streptavidin affinity chromatography followed by anti-FLAG immunoblot revealed significant proteolytic turnover of D2 receptors, as indicated by reduced biotinylated receptor signal detected in cell extracts prepared after exposure to dopamine for several hours (Fig 2C, left panel). Remarkably, dysbindin depletion visibly inhibited turnover of surface labeled D2 receptors (Fig 2C, right panel). We quantified this effect using scanning densitometry (Fig 2D) and confirmed its statistical significance across multiple independent experiments (Fig 2E).

The ability of dysbindin depletion to inhibit dopamine-induced turnover of the surface-labeled D2 receptor pool, without affecting receptor internalization itself, suggested that dysbindin regulates a later step in the endocytic pathway leading to lysosomes. To test this, we applied a previously described biochemical assay using surface biotinylation followed by cleavage by the membrane-impermeant reducing agent MESNA [14], [15], which allows stability of the internalized receptor pool to be assessed specifically. Surface-labeled receptors were completely cleaved by MESNA applied immediately after biotinylation, verifying the efficiency of the cleavage step (Fig 2F, lanes 1–2 and 5–6 from left). To assess the internalized receptor pool specifically, biotinylated cells were exposed to 10 µM dopamine for 30 min prior to cleavage of residual surface-accessible receptors by MESNA, resulting in selective labeling of the pool of receptors internalized during this time period. We then assessed the biochemical stability of this receptor pool following continued incubation with dopamine. The internalized pool of D2 receptors was almost completely proteolyzed within 4 hours in control cells transfected with non-silencing RNA duplex, whereas a clear inhibition of this proteolysis was observed in dysbindin-depleted cells (Fig 2F, compare lanes 4–5 with lanes 7–8). Together these results indicate that dysbindin depletion inhibits D2 receptor proteolysis after internalization.

### The Post-Endocytic Sorting Function of Dysbindin Is Not Restricted to Dopamine Receptors, yet Is Specific to a Subset of Endocytic Cargo

To test whether this effect of dysbindin is unique to the D2 receptor, or affects other receptors that undergo endocytic trafficking to lysosomes, we focused on the delta opioid receptor (DOR). DOR is another GPCR family member that is known to traffic to lysosomes after endocytosis in diverse cell types [16], [17], [18]. Dysbindin depletion up-regulated both total and surface-localized FLAG-DOR levels at steady state in HEK293 cells (Figs 3A and B). Further, dysbindin depletion significantly inhibited proteolytic down-regulation of FLAG-DOR. This was evident by examination of immunoblots normalized to the steady state receptor level, thereby allowing ligand-induced changes to be directly compared (Fig 3C). We also verified this using radioligand binding assay, which is an independent and readily quantified method (Fig 3D). Together these results indicate that the regulatory effect of dysbindin is not restricted to dopamine receptors, and they support the hypothesis that the primary mechanism of dysbindin-dependent regulation is via control of endocytic trafficking of receptors to lysosomes.

**Figure 3:** Dysbindin knockdown also inhibits lysosomal proteolysis of DORs. **A.** Immunoblot of FLAG-DOR immunoreactivity detected in HEK293 cell lysates (30 µg/lane) 3 days after transfection with dysbindin siRNA (DYS) compared to a non-silencing control RNA duplex (CTL), showing up-regulation of steady-state receptor number. Loading was normalized to equal total protein. **B.** Flow cytometric analysis showing that DYS knockdown significantly increases surface FLAG-DOR immunoreactivity. Methodology is the same as the experiment described in Fig 1B. **C.** Immunoblot analysis showing that dysbindin knockdown (DYS) inhibits proteolysis of FLAG-DOR induced by exposure of cells to the opioid agonist etorphine (10 µM) for 3 h compared to cells incubated in the absence of etorphine (t = 0). The immunoreactive species corresponding to the mature receptor is indicated by bracket. Loading was normalized to equivalent receptor levels at t = 0, to allow visual appreciation of differences in ligand-induced degradation. **D.** Radioligand binding analysis of FLAG-DOR down-regulation induced by the opioid peptide agonist DADLE (10 µM), showing that dysbindin depletion inhibits ligand-induced down-regulation at all time points examined. Statistical analysis of the difference between CTL and DYS conditions was carried out at the 4 hour time point, as indicated, using Student's t-test.

To further address the generality of dysbindin-dependent regulation of lysosomal trafficking, we examined the EGF receptor tyrosine kinase as a distinct class of endocytic cargo that undergoes selective trafficking to lysosomes [19] via a similar membrane pathway as DOR [20]. We focused on HeLa cells as another non-specialized human cell model that expresses dysbindin endogenously [21], and because these cells express EGF receptors at higher levels that HEK293 cells. To facilitate direct comparison, a stably transfected cell clone was prepared that also expressed FLAG-DOR. Immunoblot analysis failed to reveal any effect of dysbindin knockdown on steady state EGF receptor levels or ligand-induced EGF receptor proteolysis (Fig 4A). This lack of dysbindin depletion on EGF receptor stability was verified across multiple experiments using scanning densitometry (Fig 4B). Nevertheless, DOR degradation was significantly inhibited in the same cells (Fig. 4C).

**Figure 4:** Dysbindin knockdown inhibits FLAG-DOR proteolysis in HeLa cells, but does not affect down-regulation of EGF receptors. **A.** Immunoblot analysis of endogenous EGFRs in lysates (30 µg/lane) prepared from HeLa cells that also express FLAG-DOR (introduced by stable transfection), prepared after incubating serum-starved cells for the indicated time with 100 ng/ml EGF. **B.** Quanitification of ligand-induced proteolysis of EGFRs by scanning densitometry of immunoblots from multiple (n = 5) experiments. **C.** Quantification of ligand-induced proteolysis of FLAG-DOR in the same HeLa cell clone (n = 5). The statistical significance of the difference between CTL and DYS conditions was calculated at the 1 hour (panel B) or 3 hour (panel C) time point using Student's t-test.

### Dysbindin Promotes Connectivity of Specific Signaling Receptors to the Conserved ESCRT Machinery

The selective effect of dysbindin in promoting proteolysis of GPCRs, but not the EGFR, was reminiscent of the effect of G protein-coupled receptor-associating proteins (GASPs or GPRASPs), which are thought to modulate lysosomal trafficking of various GPCRs by direct interaction [22]. Thus we asked if GASPs might physically interact with dysbindin in intact cells. To do so, we co-expressed a GFP-tagged GASP1/GPRASP1 (GFP-GASP1) with HA-tagged dysbindin (DYS-HA) in HEK293 cells and tested association by co-immunoprecipitation. GFP-GASP1 clearly pulled down DYS-HA. We did not observe any detectable interaction with GFP alone or with GFP fused to an irrelevant protein (the PDZ domain isolated from alpha-syntrophin), even when these proteins were significantly over-expressed relative to GFP-GASP1 (Fig 5A).

**Figure 5:** Dysbindin associates with GASP1 and HRS. **A.** Co-immunoprecipitation of a GFP-tagged version of full-length GASP1 (GFP-GASP1) with DYS-HA from lysates prepared from transfected HEK293 cells. Asterisk indicates immunoreactive signal representing DYS-HA isolated in the GFP-GASP1 but not control (GFP or GFP-PDZ) immunoprecipitate. Arrow indicates GFP-GASP1 and arrowhead indicates GFP. **B.** Co-immunoprecipitation of Myc-HRS with DYS-HA from transfected HEK293 cell lysates. Asterisk indicates DYS-HA that copurified specifically with Myc-HRS but not with GFP or with Myc-HRS-ΔCC. **C.** Colocalization of DYS-GFP with a subset of endosomes labeled by Cherry-HRS. A representative image is shown and scale bar indicates 10 µm. **D.** Model for the proposed function of dysbindin in specifically promoting the post-endocytic sorting of GPCRs to lysosomes via GASP/HRS connectivity. GASP1 localizes predominantly to the cytoplasm, suggesting that it acts as a transient linker.

If dysbindin links GPCRs to the degradative pathway, we next asked if this protein may associate with core machinery mediating MVB/lysosome sorting. HRS is a component of the endosome-associated ‘ESCRT 0’ complex that mediates the initial selection of endocytic cargo for lysosome delivery [23]. HRS because is well known to be required for lysosomal sorting of ubiquitinated EGFRs [24]. HRS is similarly required for lysosomal sorting of DORs, even when receptor ubiquitination is prevented by mutation [20]. We also noted that a genome-wide yeast 2-hybrid screen identified dysbindin as an interaction partner for HRS [25]. To ask if dysbindin is capable of associating with HRS in intact cells, we again used co-immunoprecipitation analysis. Myc-tagged HRS (Myc-HRS) pulled down DYS-HA specifically, as indicated by the loss of this signal in control experiments in which Myc-HRS was replaced by GFP. Further supporting the specificity of this interaction, a mutant HRS construct missing the conserved coiled-coil domain (Myc-HRS-ΔCC) also failed to pull down DYS-HA.

We next asked if dysbindin can be observed on the same endosomal compartment with HRS. Endogenous dysbindin has been shown previously to localize to endosome membranes [26], and endosome localization of endogenous HRS is well-established [23], [24]. While we could easily detect endogenous dysbindin in HEK293 and HeLa cells by immunoblot, the reagents available to us were not suitable for immunocytochemical localization. Thus we examined the distribution of a GFP-tagged version of DYS (DYS-GFP) when co-expressed in HEK293 cells with mCherry-tagged Hrs (Cherry-HRS). DYS-GFP was observed largely in a diffuse cytoplasmic distribution, but a fraction was also localized to intracellular membranes (Fig 5C, top panel). Examination of Cherry-HRS localization in the same cells indicated that these structures represent a subset of HRS-positive endosomes (Fig 5C, middle and bottom panels).

## Discussion

In the present study we identify a role of dysbindin in promoting the post-endocytic sorting of GPCRs to lysosomes. We first observed this effect based on the study of D2 dopamine receptors, whose surface expression was significantly up-regulated at steady state in dysbindin-depleted cells. This up-regulation was consistent with the previously reported effect of dysbindin depletion in neurons [13]. Further analysis indicated that dysbindin depletion specifically inhibited lysosomal proteolysis of receptors after endocytosis, without detectably affecting ligand-induced endocytosis of receptors. This effect was not restricted to D2 receptors, as proteolytic down-regulation of another lysosomally-sorted GPCR (DOR) was also affected. Down-regulation of the EGF receptor tyrosine kinase, however, was not detectably inhibited. This selective regulation of GPCRs was reminiscent of the previously proposed role of GASPs (or GPRASPs) in modulating lysosomal sorting of both DOR and D2 (but not EGF) receptors by direct interaction [22], [27]. Further, co-immunoprecipitation analysis detected association of dysbindin with GASP1 in cell extracts. Dysbindin knockdown, in contrast to its pronounced effect on surface expression of both D2 receptors and DOR, did not detectably affect surface expression of D1 dopamine receptors. This is consistent with previous data indicating that D1 receptors preferentially recycle after endocytosis, and bind relatively poorly to GASPs [27]. Thus, taken together, the present results identify a distinct and essential role of dysbindin in promoting the lysosomal trafficking of a subset of endocytic membrane cargo after endocytosis (Fig. 5D). In further support of this we note that a recent paper, published while the present study was in review, showed that depleting dysbindin increased D2 receptor recycling in neurons [28]. Considering that the DTNBP1 gene is broadly expressed, we believe that dysbindin may play a significant role in controlling the post-endocytic sorting of various GPCRs and in multiple cell types.

An important direction for future investigation will be to further elucidate the biochemical mechanism by which dysbindin mediates its post-endocytic sorting function. The detection of co-immunoprecipitation with HRS suggests that dysbindin may function at an early step in lysosomal trafficking, by promoting indirect receptor connectivity (through GASPs) to the conserved ESCRT machinery. Dysbindin is known to assemble in a multi-protein complex (BLOC-1), and has been reported to associate with other cytoplasmic proteins as well [21], [29]. It will be interesting in future studies to investigate if any of these other components are essential for GPCR sorting to lysosomes. It will also be interesting to define the structural basis of the dysbindin-HRS association, and determine whether this interaction is essential for the observed GPCR sorting activity. Evidence of dysbindin-HRS interaction was observed previously in a yeast 2-hybrid screen [25], suggesting that dysbindin is capable of binding HRS directly.

We propose that the present observations, in additional to their basic cell biological significance, may contribute to mechanistic understanding of complex genetic diseases. Mutations in the dysbindin gene (DTNBP1) have been implicated in various human neuropsychiatric disorders characterized by disturbances in cognition, including schizophrenia. Further, a loss-of-function mutation in dysbindin produces significant neurobehavioral defects in mice [30], [31], [32]. While many studies support disturbances of D2 receptor signaling or regulation in schizophrenia, there is evidence for dysregulation of other signaling systems as well [3]. We suggest that the present results, by identifying a distinct cellular function of dysbindin that is not restricted to this particular GPCR, may provide new insight to how mutation in a single candidate gene can produce complex effects on disease vulnerability.

## Materials and Methods

### Cell Culture, cDNA Constructs, and Transfection

A Myc-tagged mouse HRS (Myc-HRS) construct was a gift from Harald Stenmark (University of Oslo) and was previously described by his group [33]. A fluorescently tagged version (Cherry-HRS) was generated by replacing the N-terminal Myc tag with mCherry using PCR. A version missing the coiled-coil domain (Myc-HRS-ΔCC) was constructed using PCR to remove amino acids 401–508 from the mouse HRS sequence. Mouse dysbindin was a generous gift from Maria Wei (UCSF) and was tagged at its C-terminus with either an HA epitope (DYS-HA) or GFP (DYS-GFP), and inserted into pIREShygro3 (Clontech). A GFP-tagged version of GASP1 (GFP-GASP1) was constructed attaching GFP to the N-terminus of the previously described human GASP1 (GPRASP-1) construct [22]. A GFP-tagged version of the conserved PDZ domain isolated from mouse alpha-1 syntrophin (residues 71–177) was used as an additional non-specific control because this construct (GFP-PDZ) is know to bind a variety of other cellular proteins. FLAG-tagged versions of the human D1 and D2 (long isoform) dopamine receptors, and the mouse delta opioid receptor have been previously described [34], [35]. Stably transfected cells expressing the indicated receptor constructs were generated by selection for neomycin resistance using 500 µg/ml G418 (Geneticin, Invitrogen). Resistant colonies were clonally isolated and selected for further study based on comparable levels of receptor expression as assessed by fluorescence microscopy. HEK293 cells (ATCC, Manassas, VA) were maintained in Dulbecco's modified Eagle's medium supplemented with 10% fetal bovine serum (University of California, San Francisco, Cell Culture Facility).

HRS and Dysbindin constructs were expressed by transient transfection using Lipofectamine 2000 (Invitrogen) according to the manufacturer's instructions. Cells expressing FLAG-tagged receptors were harvested by washing with EDTA and plated in 6 cm dishes at 80% confluence before transfection with plasmid DNA. Cells were reseeded into polylysine-coated 6-well or 24-well plates and cultured for an additional 24 h before experimentation. For knockdown of endogenous Dysbindin, the following siRNA duplexes were obtained from Qiagen: Dysbindin, DTNBP1 siRNA#1 (Hs_DNTBP1_3), r(ACU GGA GAA UUA CAA GAA A)dTdT, siRNA#2 r(AAG UGA CAA GUC AAG AGA A)dTdT, siRNA#3 Ambion: (siRNA ID# s38427) r(CAG CAA AUC UGA CUC AUU U)dTdT. The control duplex used for comparison was r(AAU UCU CCG AAC GUG UCA CG)dT. They were transfected using Lipofectamine RNAi-max (Invitrogen) using the optimized protocol provided by the manufacturer for HEK293 and HeLa cells. In all experiments reagent amounts were scaled according to surface area of the specific culture dishes used, based on the optimized protocol listed for 24-well plates. Experiments were conducted 3 days after siRNA transfection.

### Biochemical Detection of Receptors by Immunoblotting

Cell monolayers were washed three times in ice-cold phosphate-buffered saline (PBS) and lysed in extraction buffer (0.1% Triton X-100, 150 mM NaCl, 25 mM KCl, 25 mM Tris, pH 7.4) supplemented with a standard protease inhibitor mixture (Roche Applied Science). Extracts were clarified by centrifugation (20,000×g for 15 min) and then mixed with lithium dodecylsulfate (LDS) sample buffer for denaturation and 1% beta-mercaptoethanol for reduction, and incubated for 5 minutes at room temperature. Unless specified otherwise, total protein levels for each well were normalized to each other by averaging 3 measurements of Coomassie Plus in a 96 well plate reader. Proteins present in the extracts were resolved by LDS-PAGE using 4–12% BisTris gels (NuPAGE; Invitrogen), transferred to nitrocellulose membranes, and probed for tagged protein by immunoblotting using the indicated primary antibody. Horseradish peroxidase-conjugated sheep anti-mouse IgG or donkey anti-rabbit IgG (Amersham Biosciences) was used as secondary antibody, as appropriate, followed by detection of immunoreactivity using SuperSignal detection reagent (Pierce). Apparent molecular mass was estimated using commercial protein standards (SeeBlue Plus2; Invitrogen). Band intensities of unsaturated immunoblots were analyzed and quantified by densitometry using FluorChem 2.0 software (AlphaInnotech Corp.). Antibodies used (all at 1∶1000) were anti-FLAG-M1, anti-FLAG-M2-HRP (Sigma), anti-HA-11 (Covance), anti-HA(3F10)-HRP (Roche Applied Science), and Mouse Diclonal anti-GFP (Roche Applied Science). Rabbit anti-Dysbindin was a generous gift from Esteban Dell'Angelica (University of California Los Angeles), and has been previously described [36].

#### Biotinylation-Degradation Assay

Proteolysis of surface-labeled receptors was assessed using domain-specific biotinylation, as described previously [17]. Briefly, HEK293 cells expressing the indicated receptor construct were plated on 6 cm dishes, washed with ice-cold PBS, and incubated with 300 µg/ml sulfo-N-hydroxysuccinimide-biotin (Pierce) in PBS for 30 min at 4°C to selectively label proteins present in the plasma membrane. Following washing with Tris-buffered saline to remove and quench unreacted biotinylation reagent, cells were returned to 37°C and incubated in the absence or presence of 10 µM dopamine for the indicated time period, then extracted as described above. Extracts were clarified by centrifugation (20,000×g for 15 min), and biotinylated proteins were isolated by immobilization on streptavidin-conjugated Sepharose beads (Pierce). Washed beads were eluted with LDS sample buffer before resolving by SDS-PAGE, transferred to nitrocellulose membranes, and probed for FLAG-tagged receptor (M1 antibody; Sigma).

### Biotin Protection/Degradation Assay

HEK293 cells stably expressing FLAG-D2 receptors were grown to 100% confluency in 10-cm plates and subjected to the biotin protection/degradation assay protocol as described previously [14], [15]. Cells were left untreated or stimulated for 1 hour or 4 hours with 10 µM dopamine for the same times indicated. Briefly, cells were treated with 3 µg/ml disulfide-cleavable biotin (Pierce) for 30 min at 4°C. Cells were then washed in PBS and placed in prewarmed conditioned medium for 15 min before treatment with ligand (or no treatment) for 30 minutes to allow for internalization. Concurrent with ligand treatment non-strip and strip plates remained at 4°C. After ligand treatment for 30 minutes, plates were washed in PBS, and remaining cell surface-biotinylated receptors were stripped 3× in 100 mM MESNA, 50 mM Tris, 100mM NaCl, 1mM EDTA, and 0.2% BSA at 4°C for 15 minutes. Cells were quenched with PBS containing 120 mM iodoacetamide, 1% bovine serum albumin and then incubated with agonist for the indicated time period. The cells were then lysed in 0.1% Triton X-100, 150 mM NaCl, 25 mM KCl, 10 mM Tris·HCl, pH 7.4, with protease inhibitors (Roche Applied Science, Basel, Switzerland). Lysates were cleared at 20,000 g for 15 minutes and then precipitated with streptavidin beads (Pierce), and resolved by LDS-PAGE, transferred to nitrocelluse and finally probed for receptor with anti-FLAG-M2-HRP.

#### Analysis of Receptor Number and Ligand-Induced Down-Regulation by Radioligand Binding

Down-regulation of FLAG-DOR expressed in stably transfected HEK293 cells was determined by radioligand binding, using the radiolabeled antagonist [3H]diprenorphine (DPN) (88 Ci/mmol; Amersham Biosciences) exactly as previously described [37]. Nonspecific binding was determined by carrying out parallel determinations in the presence of excess unlabeled competitive antagonist (10 µM naloxone). Data presented represent the specific binding (total minus nonspecific binding) at each time point, expressed as a percentage of specific binding in similarly transfected but agonist-naive cells.

#### Fluorescence Microscopy

Colocalization of Dysbindin-GFP with mCherry-HRS was visualized in HEK293 cells plated on polylysine-coated glass coverslips (Corning Glass). Cells were fixed 2 days post transfection with 3.7% formaldehyde and permeabilized with 0.1% Triton X-100 in PBS. Specimens were imaged by confocal fluorescence microscopy using a Zeiss LSM 510 microscope fitted with a Zeiss ×63, numeric aperture 1.4 objective operated in single photon mode, with standard filter sets verified for lack of detectable cross-channel bleed-through and standard (1 Airy disc) pinhole. Acquired optical sections were analyzed with LSM Image Examiner (Zeiss) and rendered with Adobe Photoshop software.

### Fluorescence Flow Cytometry

Surface receptor immunoreactivity was assayed by incubating intact, non-permeabilized cells with Alexa647-conjugated anti-FLAG M1 antibody (1 µg/ml for 45 min), washed, and analyzed by fluorescence flow cytometry using a FACSCaliber instrument (Becton Dickenson). For each condition, staining was performed in triplicate and 10,000 cells per tube were were analyzed. Intensity values were determined using the geometric mean.

#### Statistical Analysis

Quantitative data were averaged across multiple independent experiments, with the number of experiments specified in the corresponding figure legend. Unless indicated otherwise, the error bars represent the S.E.M. calculated across experiments. The statistical significance of the indicated differences was analyzed using Student's t test, calculated using Prism 4.0 software (GraphPad Software, Inc.).
